The article "MircoRNA-33a inhibits epithelial-to-mesenchymal transition and metastasis and could be a prognostic marker in non-small cell lung cancer" was retracted in 2021. Reasons: duplicated images; unreliable data.

# MircoRNA-33a inhibits epithelial-to-mesenchymal transition and metastasis and could be a prognostic marker in non-small cell lung cancer

**DOI:** 10.1038/srep13677

**Published:** 2015-09-02

**Authors:** Lihua Yang, Jie Yang, Jingqiu Li, Xingkai Shen, Yanping Le, Chengwei Zhou, Shaomin Wang, Shun Zhang, Dazhi Xu, Zhaohui Gong

**Affiliations:** 1 Institute of Biochemistry and Molecular Biology; 2 Zhejiang Provincial Key Laboratory of Pathophysiology, Ningbo University School of Medicine, Ningbo, ZJ 315211, China; 3 Department of Chest Surgery; 4 Department of Oncology, The Affiliated Hospital of Ningbo University School of Medicine, Ningbo, ZJ 315020, China; 5 Clinical Laboratory, Ningbo No. 2 Hospital, Ningbo, ZJ 315010, China; 6 State Key Laboratory of Oncology in South China; 7 Sun Yat-sen University Cancer Center, Guangzhou, GD 510060, China

## Abstract

Understanding the molecular mechanism by which epithelial mesenchymal transition (EMT)-mediated cancer metastasis and how microRNA (miRNA) regulates lung cancer progression via Twist1-activated EMT may provide potential therapeutic targets for cancer therapy. Here we found that miR-33a, an intronic miRNA located within the sterol regulatory element-binding protein 2 (SREBP-2) gene, is expressed at low levels in metastatic non-small cell lung cancer (NSCLC) cells and is inversely correlated with Twist1 expression. Conversely, miR-33a knockdown induces EMT and miR-33a overexpression blocks EMT by regulating of Twist1 expression in NSCLC cells. Bioinformatical prediction and luciferase reporter assay confirm that Twist1 is a direct target of miR-33a. Additionally, Twist1 knockdown blocks EMT-related metastasis and forced expression of miR-33a inhibits lung cancer metastasis in a xenograft animal model. Clinically, miR-33a is found to be at low levels in NSCLC patients and down-regulation of miR-33a predicts a poor prognosis. These findings suggest that miR-33a targets Twist1 and inhibits invasion and metastasis in NSCLC. Thus, miR-33a might be a potential prognostic marker and of therapeutic relevance for NSCLC metastasis intervention.

Distant metastasis causes more than 90% of non-small cell lung cancer (NSCLC) deaths and is a complex series of steps in which cancer cells leave the original tumor site and migrate to other parts of the body via the bloodstream and the lymphatic system^1^. A cell-biological program called the epithelial to mesenchymal transition (EMT) is a fundamental process and a key step toward cancer metastasis^2^. The completion of EMT is signaled by the degradation of the underlying basement membrane and the formation of a mesenchymal cell that can migrate away from the epithelial layer from which it originates^3^. EMT not only occurs in embryonic development but also contributes to various pathological conditions^4^. Recent studies show that many transcription factors are involved in EMT, such as Twist1^5^. However, the regulatory mechanism for Twist1-related EMT in NSCLC metastasis remains poorly understood.

The article "MircoRNA-33a inhibits epithelial-to-mesenchymal transition and metastasis and could be a prognostic marker in non-small cell lung cancer" was retracted in 2021. Reasons: duplicated images; unreliable data.

MicroRNAs (miRNAs), as a class of small and non-coding RNAs, play important roles in a great many biologic processes^6^. Increasing bodies of evidences demonstrate that miRNAs can act as oncogenes or tumor suppressors and regulate cancer cell metastasis^7^,^8^,^9^. MiR-33a, an intronic miRNA located within the sterol regulatory element-binding protein 2 (SREBP-2) gene, was originally found to regulate cholesterol metabolism^10^,^11^, and then to control cell cycle^12^,^13^. A given miRNA may represent pleiotropic effects on cellular functions, whether miR-33a is directly involved in EMT and metastasis in NSCLC has not been reported.

Although miRNAs may act as critical regulators in cancer metastasis, the mechanism how miR-33a regulates metastasis by targeting the EMT-relevant transcriptional factors was unknown at the onset of this study. Here, we provide the first demonstration that miR-33a modulates EMT in NSCLC cells and targets Twist1, an EMT-inducing transcription factor. Furthermore, miR-33a suppresses NSCLC metastasis *in vivo* in a xenograft mouse model. Our findings suggest that miR-33a could be used as a potential therapeutic RNA mimic (miRNA replacement) for the treatment of patients with the advanced NSCLC.

## Results

### miR-33a is expressed at low levels in metastatic NSCLC cells

To investigate the migratory capability of NSCLC cells, the wound healing assay was performed. Among the tested cell lines, NCI-H1299 cells migrated the longest distance that showed a high metastasis rate, whereas SPC-A-1 cells migrated the shortest distance that indicated a low metastasis potential (Fig. 1A). In addition, the morphology of the cells was analyzed under a phase contrast microscope. The results showed that NCI-H1299 cells exhibit a mesenchymal property as compared to the epithelial SPC-A-1 cells (Supplementary Fig. 1). Thus, we designated NCI-H1299 as a high- and SPC-A-1 as a low-metastasis cell line.

Furthermore, we determined the expression levels of miR-33a in these cell lines. The real-time quantitative RT-PCR analysis revealed that miR-33a was expressed at a more than 300-fold higher level in the low-metastasis SPC-A-1 cell line compared with the high-metastasis NCI-H1299 cell line (*P* < 0.001, Fig. 1B). These results indicate that miR-33a expression is strongly down-regulated in the high-metastasis cell line.

The article "MircoRNA-33a inhibits epithelial-to-mesenchymal transition and metastasis and could be a prognostic marker in non-small cell lung cancer" was retracted in 2021. Reasons: duplicated images; unreliable data.

### miR-33a is involved in EMT- dependent metastasis

To determine whether miR-33a is directly involved in EMT-dependent metastasis, the effect of miR-33a on cell EMT property was examined. The expression of miR-33a was down-regulated by the transfection of miR-33a inhibitors into the low-metastasis SPC-A-1 cell line, which expresses a relatively high level of endogenous miR-33a (Fig. 2A). In the high-metastasis NCI-H1299 cell line, the transfection of a miR-33a mimic resulted in miR-33a overexpression compared with the control RNA treatment (Fig. 2B). The results of Western blotting showed that the knockdown of miR-33a induced a marked decrease of the epithelial cell biomarker E-cadherin (CDH1) and an increase of the mesenchymal cell biomarker Vimentin (Fig. 2C), which indicated that cells had undergone an EMT. Additionally, miR-33a knockdown promoted cell migration (Fig. 2E) and invasion (Fig. 2G) in SPC-A-1 cells. In contrast, miR-33a replacement in NCI-H1299 cells increased the expression of the epithelial cell biomarker of CDH1 and decreased the expression of the mesenchymal cell biomarker Vimentin (Fig. 2D), which indicated a block of EMT. In addition, miR-33a overexpression reduced the migration (Fig. 2F) and invasion (Fig. 2H) capability of NCI-H1299 cells. Thus, the data show that miR-33a is a crucial mediator of EMT and metastasis in NSCLC cells.

### miR-33a is specifically and inversely correlated with Twist1 expression

In an effort to elucidate the mechanism of the suppression of EMT and metastasis by miR-33a, we predicted 417 potential targets for miR-33a using the TargetScan tool (http://www.targetscan.org). To further narrow down the list of potential targets, another prediction tool (http://www.microrna.org) was used. Among these candidates, Twist1 (NM_000474) was the only EMT-inducing gene. Thus, we investigated the effect of miR-33a on Twist1 gene expression. In the low-metastasis SPC-A-1 cell line, the quantitative RT-PCR and Western blot analyses indicated that miR-33a knockdown resulted in an increase in Twist1 expression at both the mRNA and protein levels (Fig. 3A,C,E). In contrast, miR-33a overexpression in NCI-H1299 cells resulted in a decrease of Twist1 gene expression (Fig. 3B,D,F). Similarly, the endogenous transcript level of Twist1 in response to miR-33a was rescued when miR-33a was cotransfected with the miR-33a inhibitor (Supplementary Fig. 2). As Pim-1, another target of miR-33a, is up-regulated in NSCLC cells and down-regulation of Pim-1 by miR-33a may contribute to the invasion and metastasis *in vitro*^12^,^14^, we compared the Pim-1 levels in NCI-H1299 cells with and without miR-33a replacement, and in SPC-A-1 cells with and without anti-miR-33a. Unfortunately, transfection of miR-33a mimics provided no evidence for a significant down-regulation of Pim-1 in NCI-H1299 cells (Supplementary Fig. 3A). Meanwhile, inhibition of miR-33a did not result in an obvious change of Pim-1 in SPC-A-1 cells (Supplementary Fig. 3B). These results indicated miR-33a negatively regulates Twist1 expression, but not Pim-1 in these two tested NSCLC cell lines. In other words, miR-33a expression is specifically and inversely correlated with Twist1 expression in NSCLC cells.

The article "MircoRNA-33a inhibits epithelial-to-mesenchymal transition and metastasis and could be a prognostic marker in non-small cell lung cancer" was retracted in 2021. Reasons: duplicated images; unreliable data.

### Twist1 is a direct target of miR-33a

To obtain the evidence that miR-33a directly regulates Twist1, we performed a luciferase reporter assay. The 3′-UTR of the human Twist1 mRNA harbors a conserved putative miR-33a binding site (Fig. 4A). The wild-type of the Twist1 3′UTR and a mutant of this sequence without the 6-nt sequence complementary to miR-33a (namely 3′UTR MUT) were cloned downstream of the *Renilla* luciferase gene (Fig. 4A,B). In the low-metastasis cell line SPC-A-1, a significant increase in the relative luciferase activity was detected when the miR-33a inhibitors were co-transfected with the wild-type construct, but not with the mutant Twist1 3′UTR (*P* < 0.001, Fig. 4C). Also in NCI-H1299 cells, a significant decrease in the relative luciferase activity was observed when the miR-33a mimic was co-transfected with the wild-type construct, but not with the mutant Twist1 3′UTR (*P* < 0.001, Fig. 4D). The data show that miR-33a directly interacts with the predicted target sequence in the Twist1 mRNA. To further investigate whether miR-33a mediates EMT phenotypes by targeting Twist1, the rescue experiment using a form of Twist1 resistant to miR-33a was performed. Interestingly, the inhibition of Twist1 overcame the increase of migration (Fig. 4E vs. Fig. 2E) and invasion (Fig. 4G vs. Fig. 2G) induced by miR-33a knockdown in SPC-A-1 cells. Similarly, the enforced expression of Twist1 rescued the decrease of migration (Fig. 4F vs. Fig. 2F) and invasion (Fig. 4H vs. Fig. 2H) mediated by miR-33a overexpression in NCI-H1299 cells. Together, these results indicate that miR-33a mediates EMT by regulating its target of Twist1.

### Twist1 knockdown blocks EMT and metastasis *in vitro*

To verify that miR-33a regulates EMT by targeting Twist1, we further investigated the role of Twist1 in EMT and metastasis. The Western blotting results showed that inhibition of Twist1 by siRNA induced the expression of CDH1 and suppressed the expression of Vimentin (Fig. 5A), which indicates a suppression of EMT. The further wound healing experiment and transwell invasion assay exhibited that Twist1 knockdown leads to the inhibition of cell migration (Fig. 5B) and invasion (Fig. 5C) in the NCI-H1299 cells. In other words, the results demonstrate that the Twist1 siRNA inhibits EMT and consequently reduces the cellular metastatic phenotype. Collectively, these results might explain the regulatory mechanism through which miR-33a represses EMT, that most likely involves the inhibition of Twist1.

The article "MircoRNA-33a inhibits epithelial-to-mesenchymal transition and metastasis and could be a prognostic marker in non-small cell lung cancer" was retracted in 2021. Reasons: duplicated images; unreliable data.

### miR-33a inhibits lung cancer metastasis in a xenograft animal model

To validate the effect of miR-33a on tumor metastasis, an *in vivo* metastasis assay was performed in severe combined immunodeficiency (SCID) mice. NCI-H1299 cells that stably expressed miR-33a and luciferase (miR-33a/luc) were injected into SCID mice via the tail vein. Cells transfected with a vector only expressed luciferase reporter were used as controls (Vec/luc). Four weeks later, the real-time *in vivo* imaging of tumors showed a significant decrease of the luciferase fluorescence signal from lung and brain in miR-33a/luc mice compared with the control (*P* < 0.001, Fig. 6A). After tested mice were sacrificed, the metastatic modules formed on the lung were counted. As shown in Fig 6B, the number of pulmonary metastatic nodules induced by miR-33a/luc cells was significantly lower than that induced by control cells (3.40 ± 1.27 versus 10.70 ± 2.21, *P* < 0.001). Further histological study with H&E stained paraffin block sections revealed that the metastatic cancers induced by miR-33a/luc cells could be only found in lung and brain, but not in other organs such as liver and uterus where metastatic cancers formed in animals injected with Vec/luc control cells (Fig. 6C). These results indicated that miR-33a inhibits *in vivo* lung tumor metastasis.

### Low miR-33a expression predicts poor prognosis in NSCLC patients

To further investigate the clinical significance of miR-33a expression in NSCLC patients, the expression levels of miR-33a were measured using qRT-PCR analysis and the survival curves were calculated by the Kaplan-Meier method. The influence of each variable on survival was examined by the Cox multivariate regression analysis. Compared with non-tumor tissues, the expression level of miR-33a was significantly decreased in NSCLC tissues (2.07 ± 0.08 versus 6.79 ± 0.12, *P* < 0.001, Fig. 7A). The expression level of miR-33a was positively correlated with grade (*P* = 0.002, Supplementary Table S1). In addition, NSCLC patients with advanced histologic grade (local invasion T3-4) had obvious shorter overall survival (OS) than patients with low grade (T1-2) (*P* = 0.0227, Fig. 7B). A significant difference was that NSCLC patients with high miR-33a expression level had remarkable longer OS than patients with low miR-33a expression level (*P* = 0.0023, Fig. 7C). Furthermore, we found that low miR-33a expression (*P* = 0.008) and advanced histologic grade (*P* = 0.004) were independent prognostic parameters indicating poor prognosis for NSCLC patients (Supplementary Table S2). Our results show that the decreased expression of miR-33a may be associated with malignant tumor progression and poor prognosis in NSCLC patients, suggesting that miR-33a may be a novel and valuable marker for predicting the clinical outcome of NSCLC patients.

The article "MircoRNA-33a inhibits epithelial-to-mesenchymal transition and metastasis and could be a prognostic marker in non-small cell lung cancer" was retracted in 2021. Reasons: duplicated images; unreliable data.

## Discussion

A given miRNA may have multiple target genes that are involved in lung cancer progression; however, most of the details of the EMT-dependent metastatic mechanism have not been elucidated. In the previous study, we revealed that miRNA could regulate lung cancer cell growth, proliferation^15^,^16^,^17^ and cisplatin-induced apoptosis^18^. The transcription factor Twist1 and the EMT-associated miRNAs are reported to be associated with cancer metastasis^19^,^20^. Here we demonstrate that miR-33a represses metastasis through targeting the EMT-associated Twist1.

Although the miR-33a dysregulation has been found in metabolism and metabolic diseases, suggesting that it might be a possible target for the treatment of cardiovascular and metabolic disorders, the effect of miR-33a on EMT and metastasis is largely unknown. Expression of miR-33a was detected in various NSCLC cells including A549, SPC-A-1, NCI-H1299, Calu-1 and NCI-H460, also revealing the interesting result that miR-33a is expressed at low levels in the high-metastasis cell line NCI-H1299, indicating that miR-33a may be associated with lung cancer metastasis. Compared with the high-metastasis cell line NCI-H1299 and the low-metastasis cell line SPC-A-1, the other three cell lines showed similar intermediate miR-33a levels, but had different metastatic potential. This phenomenon points to cell context differences of the tested cell lines. Recent studies demonstrated that miRNAs may function as “metastamiR” or “metastasis-suppressing miR”^21^,^22^. Increasing evidence indicates that EMT can be regulated by miRNAs, of which miR-34 and the miR-200 family which can promote the mesenchymal-epithelial transition (MET) and reduce tumor cell migration are mostly studied^23^. Moreover, the transcription factors and miRNAs are linked by several feedback loops. One is the double-negative feedback loop between ZEB1/2 and the miR-200 family (miR-200a, miR-200b, miR-200c, miR-141 and miR-429), in which ZEB1/2 represses the expression of miR-200 while miR-200 negatively regulates the translation of ZEB1/2^24^,^25^. Another double-negative feedback loop occurs between SNAIL and miR-34a/b/c in a similar way^26^,^27^. Also by targeting SNAI1 and ZEB2, miR-153 is a novel regulator of EMT and indicates its potential therapeutic value for reducing cancer metastasis^28^. Another miRNA, miR-148a, may negatively regulate Met/Snail signaling and therefore inhibits the EMT and metastasis of hematoma cells^29^. All of these observations indicate that miRNAs can regulate cancer metastasis through EMT. However, these functional studies have only addressed a small fraction of miRNAs. Here we focus on miR-33a, which is revealed to be involved in cell differentiation and cell polarity^30^. MiR-33a mimics decelerated tumor cell proliferation and worked as a potential tumor suppressor through inhibition of Pim-1^12^. In addition, miR-33a was also down-regulated in lung cancer cells and targeted parathyroid hormone related protein (PTHrP) to suppress bone metastasis^31^. The miRNA replacement therapy for miR-145 and miR-33a was efficacious in the colon carcinoma model^32^. In lung cancer cells, miR-33a has already been shown to directly target a potent pro-metastatic/pro-EMT gene, high mobility group AT-hook 2 (HMGA2)^33^, and this interaction is important to the anti-metastatic cellular phenotypes conferred by miR-33a. In view of our study identifying a second pro-metastatic/pro-EMT gene, Twist1, as a direct target of miR-33a, it is logical to suggest that two or more genes are employed to mediate the anti-metastatic function of miR-33a in lung cancer. Here we have provided evidence that miR-33a binds to the 3′UTR of Twist1 mRNA to suppress EMT and metastasis.

The article "MircoRNA-33a inhibits epithelial-to-mesenchymal transition and metastasis and could be a prognostic marker in non-small cell lung cancer" was retracted in 2021. Reasons: duplicated images; unreliable data.

It is well known that Twist1 belongs to the family of basic helix-loop-helix transcription factors originally found to modulate the expression of various target genes through canonical E-box responsive elements^34^. Twist1 is overexpressed in various human cancers^35^,^36^,^37^ including lung cancer. Evidences also indicate that Twist1 contributes to cancer cell dissemination by promoting EMT and increasing cellular invasiveness^38^,^39^, and also induces endothelial differentiation of cancer cells^40^. Twist1 is regulated by some miRNAs (miR-720^41^, miR-106b^42^ and miR-675^43^) and finally affects tumor metastasis. Interestingly, Twist1 also regulates miRNA expression. miR-10b transcription is directly regulated by Twist1, and miR-10b in turn inhibits translation of the mRNA encoding homebox D10, resulting in the increased expression of the pro-metastatic gene RhoC. Moreover, the level of miR-10b expression in primary breast carcinomas is associated with clinical cancer progression^44^. These findings mean that Twist1 indirectly up-regulates RhoC expression to promote breast cancer cell invasion and metastasis.

The article "MircoRNA-33a inhibits epithelial-to-mesenchymal transition and metastasis and could be a prognostic marker in non-small cell lung cancer" was retracted in 2021. Reasons: duplicated images; unreliable data.

In conclusion, our study has shown that the up-regulation of miR-33a blocks EMT and metastasis. We further demonstrate that miR-33a regulates EMT by targeting Twist1 in NSCLC cells and inhibits lung cancer metastasis. Thus, increasing the cellular levels of miR-33a may be a novel therapeutic strategy for the treatment of patients with advanced NSCLC.

## Methods

### Cell culture and transfection

A549 and NCI-H460 cells were cultured in RPMI-1640 medium (Invitrogen, USA) supplemented with 1.5 g/L sodium bicarbonate and 10% fetal bovine serum (FBS) (Hyclone, USA). NCI-H1299 and SPC-A-1 cells were maintained in RPMI 1640 containing 1 mM pyruvic acid sodium, 4.5 g/L glucose, 1.5 g/L sodium bicarbonate and 10% FBS. Calu-1 cells were cultured in McCoy’s 5A (Sigma, Germany) supplemented with 10% FBS and 1.5 g/L sodium bicarbonate. All of the cells were cultured at 37 °C in a humidified atmosphere containing 5% CO_2_. The logarithmically growing cells were transfected with miR-33a (mimics) and its corresponding control RNA (mimics NC), or anti-miR-33a (inhibitors) and its corresponding control RNA (inhibitor NC), or Twist1 siRNA (siTwist1) (GenePharma, China) as previously described^18^. The sequences of the miRNA and siRNA oligonucleotides are shown in supplementary Table 3.

### Patients and tissue specimens

We studied the specimens of tumor tissue and its matching normal tissue from 53 patients who underwent surgical resection of NSCLC at the Affiliated Hospital of Ningbo University School of Medicine. The patients had not received adjuvant chemotherapy. According to WHO criteria, 53 NSCLC patients were classified as low-grade (I–II) and high-grade (III–IV). All patients were under a close follow-up observation for disease recurrence at no less than 3-month intervals during the first two postoperative years, and no less than every 6 months thereafter. Overall survival (OS) time was calculated from the date of the initial surgery to death. This study was carried out in accordance with the approved guidelines by the Medical Ethical Committee at Ningbo University. Written informed consent was obtained from all patients.

### Real-time RT-PCR

The total RNAs from the transfected cells or tumor tissues were isolated using RNAiso Plus (Takara, Japan). One microgram of total RNA was subjected to a reverse transcription reaction. For the miR-33a quantification, real-time quantitative PCR of miR-33a was performed on a Mx3005P system (Stratagene, USA) using the Hairpin-it^TM^ miR qPCR quantification kit (GenePharma, China) and the SYBR Premix ExTaq II reagent (Takara, Japan). The reaction was performed in an 8-strip tube under the following conditions: 95 °C for 2 min, 40 cycles of 95 °C for 20 s, 60 °C for 1 min, and 72 °C for 1 min, and a final extension at 72 °C for 5 min. The E-cadherin, Vimentin and Twist1 were normalized to that of the housekeeping gene β-actin as an endogenous control. The primer sequences used for real-time RT-PCR analyses are shown in supplementary Table 4.

The article "MircoRNA-33a inhibits epithelial-to-mesenchymal transition and metastasis and could be a prognostic marker in non-small cell lung cancer" was retracted in 2021. Reasons: duplicated images; unreliable data.

### Cell lysates and Western blotting

Whole-cell lysates were prepared in RIPA buffer(50 mM Tris-HCl pH8.0, 150 mM NaCl, 1%Triton X-100, and 1 protease inhibitor cocktail tablet/10 ml), and the Western blotting was performed as previously described^18^. The primary antibodies used were E-cadherin (CST, USA), Vimentin (CST, USA), Twist1 (Sigma, USA), Pim-1 (SantaCruz, USA) and β-actin (HuaAn, China).

### Migration and invasion assays

The capability of tumor cell migration was assessed using a wound-healing assay. Confluent cell monolayers were manually wounded by scraping the cells with a 200 μl pipette tip. Photos were taken at 0, 24, 48 h. The distances were assessed by Image-Pro Plus 6.0 software.

For invasion assays, infected or transfected cells were harvested and resuspended in serum-free RPMI-1640 medium, and 1 × 10^5^ cells were placed into chambers coated with 150 μg of Matrigel (BD Bioscience, USA). The chambers were then inserted into the wells of a 24-well plate and incubated for 48 h in RPMI-1640 medium with 20% fetal bovine serum before examination. The cells remaining on the upper surface of the membranes were removed, whereas the cells adhering to the lower surface were fixed, stained in a dye solution containing 0.05% crystal violet (Solarbio, China) and the stained cells were resolved by 30% acetic acid and OD_570_ was measured by Spectramax M5 (Molecular Devices, USA).

### Plasmid construction

The predicted miR-33a binding site in the 3′UTR of Twist1 gene was cloned downstream of the firely luciferase gene as follows: cDNA from NCI-H1299 cells was amplified by PCR using specific primers (shown in supplementary Table 4) for Twist1 cloning. The PCR product was then digested with *Xba* I and inserted into the *Xba* I site of the pGL3 control vector (Promega, USA), after sequencing confirmation, the new combined plasmid was designated as pGL3-Twist1-WT. The mutation of the 3′UTR of Twist1 was also achieved like that and named pGL3-Twist1-MUT after sequencing. For construction of pcDNA-Twist1, the full-length cDNA of Twist1 was obtained by RT-PCR using gene-specific primers (shown in supplementary Table 4) and subcloned into *BamH* I and *EcoR* I sites of the pcDNA3.1 vector.

### Luciferase reporter assays

The SPC-A-1 and NCI-H1299 cells were seeded in 6-well plates (1 × 10^5^ cells/well) and incubated for 24 h before transfection. For reported gene assay, the cells were contransfected with 1ug of pGL3-Twist1-3′UTR or pGL3-Twist1-3′UTR MUT plasmid, 0.5 ug of the phRL-SV40 control vector (Promega, USA). The firely and *Renilla* luciferase activities were measured consecutively through a dual luciferase assay (Promega, USA) 24 h after transfection.

The article "MircoRNA-33a inhibits epithelial-to-mesenchymal transition and metastasis and could be a prognostic marker in non-small cell lung cancer" was retracted in 2021. Reasons: duplicated images; unreliable data.

### Animal experiments

The experiments were performed in accordance with the approved guidelines by the Laboratory Animal Ethical Committee at Ningbo University. NCI-H1299 cells stably overexpressing miR33a and luciferase (miR-33a/luc) were constructed by using a lentivirus-based method as previously described^45^. Then SCID mice were intravenously inoculated with NCI-H1299 cells expressing miR-33a/luc or the control cells (Vec/luc) to construct NSCLC xenograft models. Using an *in vivo* imaging system (Korda, USA), we monitored the growth and metastasis of the tumors. Finally, we verified the extents of tumorigenesis and metastasis by tissue sections with hematoxylin and eosin (H&E) staining.

### Statistical analysis

The data were assessed using the Graphpad Prism 5.0 software (Graphpad, USA). All of the experiments were performed in triplicate, and Student’s t-test was used to analyze the significance of the difference levels between two groups. The expression of miR-33a was assessed for associations with clinicopathological factors using Chi-square test. The survival curves were calculated by the Kaplan-Meier method and the difference by the Log-rank test. The influence of each variable on survival was examined by the Cox multivariate regression analysis. The statistical significance was set to *P* < 0.05 in each test.

## Additional Information

**How to cite this article**: Yang, L. *et al.* MircoRNA-33a inhibits epithelial-to-mesenchymal transition and metastasis and could be a prognostic marker in non-small cell lung cancer. *Sci. Rep.* **5**, 13677; doi: 10.1038/srep13677 (2015).

## Supplementary Material

Supplementary Information

## Figures and Tables

**Figure 1:** miR-33a is low-expressed in metastatic cell lines. (**A**) Identification of different metastatic potent of NSCLC cell lines. The distance after 12 h is shown. (**B**) Basal expression of miR-33a in NSCLC cell lines. The data present the levels of mature miR-33a relative to that in NCI-H1299 cells. ***P < 0.001.

**Figure 2:** miR-33a knockdown induces EMT and metastasis and miR-33a overexpression blocks EMT and metastasis. (**A**) SPC-A-1 cells was transfected with miR-33a inhibitors (anti-miR-33a) or inhibitor NC (Ctrl RNA) and (**B**) NCI-H1299 cells was transfected with miR-33a mimics (miR-33a) or mimics NC (Ctrl RNA), the levels of mature miR-33a were confirmed by quantitative RT-PCR. Western Blotting was performed after the transfection of RNAs. The changes of epithelial cell biomarker E-cadherin and mesenchymal cell biomarker Vimentin were shown in SPC-A-1 (**C**) and NCI-H1299 (**D**) cells. The migration and invasion capability were respectively measured after the transfection of RNA oligos in SPC-A-1 (**E**,**G**) and NCI-H1299 (**F**,**H**) cells. *P < 0.05, **P < 0.01, ***P < 0.001.

The article "MircoRNA-33a inhibits epithelial-to-mesenchymal transition and metastasis and could be a prognostic marker in non-small cell lung cancer" was retracted in 2021. Reasons: duplicated images; unreliable data.

**Figure 3:** miR-33a negatively regulates Twist1 expression. Quantitative RT-PCRs of Twist1 mRNA expressions in SPC-A-1 and NCI-H1299 cells were performed after transfections of anti-miR-33a (**A**) and miR-33a (**B**). Western blotting (**C**,**D**) and semi-quantitative analyses (**E**,**F**) of Twist1 protein in SPC-A-1 and NCI-H1299 cells treated as described above. *P < 0.05, **P < 0.01.

**Figure 4:** Twist1 is a direct target of miR-33a. (**A**) Predicted the binding site of miR-33a in Twist1 3′UTR that is complementary to miR-33a. (**B**) The sequences of the wild-type (top) and the mutant (bottom) Twist1 3′UTR used for the dual-luciferase reporter construct. (**C**) miR-33a knockdown promotes the wild-type Twist1 3′UTR reporter but not the mutant Twist1 3′UTR reporter in SPC-A-1 cells. (**D**) miR-33a inhibits the wild-type Twist1 3′UTR reporter but not the mutant Twist1 3′UTR reporter in NCI-H1299 cells. The migration and invasion capability were separately measured after the transfections of RNA oligos and plasmids in SPC-A-1 (**E**,**G**) and NCI-H1299 (**F**,**H**) cells. ***P < 0.001.

**Figure 5:** Twist1 knockdown blocks EMT and metastasis. NCI-H1299 cells subjected to Twist1 siRNA knockdown and Western blotting was performed after 48h. The changes of epithelial cell biomarker E-cadherin and mesenchymal cell biomarker Vimentin and the semi-quantitative analyses were shown (**A**). The migration (**B**) and invasion (**C**) capability were measured after transfections of siRNA. *P < 0.05, **P < 0.01, ***P < 0.001.

**Figure 6:** miR-33a inhibits tumor metastasis in xenograft mouse model. (**A**) Real-time *in vivo* imaging showed the tumor metastasis post-intravenous injection of miR-33a/luc or Vec/luc cells by tail vein (left), the luciferase fluorescence values were compared between these two groups (right, n = 10 in each group). (**B**) The pulmonary metastatic nodules were counted (left) and compared in the sacrificed mice (right, n = 10). (**C**) The metastatic cancer tissues (lung, brain, liver and uterus) were confirmed by H&E staining. ***P < 0.001.

**Figure 7:** Low-expression of miR-33a predicts poor prognosis in NSCLC patients. (**A**) Relative miR-33a expression levels were measured in 53 pairs of NSCLC tumor and non-tumor tissue samples by real-time quantitative RT-PCR. (**B**) The association of local invasion and overall survival in NSCLC patients. (**C**) The expression level of miR-33a in relation to overall survival in NSCLC patients. ***P < 0.001.
